The article "Exploring the Potential of Interferon Gamma Gene as Major Immune Responder for Bovine Tuberculosis in River Buffalo" was retracted in 2024. Reasons: signs of a paper mill; suspected computer-generated content; unreliable results or conclusions; concerns about the data.

# Exploring the Potential of Interferon Gamma Gene as Major Immune Responder for Bovine Tuberculosis in River Buffalo

**DOI:** 10.1155/2021/5532864

**Published:** 2021-04-05

**Authors:** Maryam Javed, Syed Ahmed Raza, Asif Nadeem, Muhammad Muddassir Ali, Wasim Shehzad, Khalid Mehmood

**Affiliations:** ^1^Institute of Biochemistry and Biotechnology, University of Veterinary and Animal Sciences, Lahore, Pakistan; ^2^Department of Biotechnology, Virtual University of Pakistan, Lahore, Pakistan; ^3^Faculty of Veterinary and Animal Sciences, The Islamia University of Bahawalpur, 63100, Pakistan

## Abstract

Bovine tuberculosis (bTB) is a widespread zoonotic infection targeting the livestock sector, especially in developing countries, and posing a risk to humans and animal populations. Its recent prevalence in river buffaloes has been estimated as higher as 33.7%. In emergent countries like Pakistan, there is likeliness of human-livestock interfaces extensively and lacking of effective preventive measures that illustrate the risk of spreading the infection at a remarkable rate. The river buffalo (*Bubalus bubalis*) is an upkeep host of *Mycobacterium bovis* and is responsible for disease transmission among buffaloes and other livestock species. In this study, potential molecular biomarkers in the Interferon-gamma gene (IFNg) were identified after genomic screening of river buffaloes. Unique genomic loci in river buffalo proved the novelty of the genomic structure of this phenomenal animal but also highlighted its significance in natural immunity against the *Mycobacterium*. A total of eight single nucleotide polymorphisms were identified in the coding region of IFNg. The SNPs in the exonic region were all transitions, i.e., the conversion of purines to purines. These SNPs were analyzed for Hardy Weinberg Equilibrium, chi^2^ test, gene diversity, and protein structural conformation. Pathway analysis in tuberculosis revealed that IFNg inhibits the antigen-presenting cells (APC) through JAK and STAT pathways. Network analysis of IFNg proteins in both species showed strong associations among the immunity-related proteins (interleukins, tissue necrosis factors) and receptors of interferons. The identified polymorphic sites might be novel-potentiated markers for the selection of animals with superior immune response against bTB and can be exploited as promising genomic sites for breeding the resistant animal herds to combat *Mycobacterium* infection in a long run.

## 1. Introduction

Bovine tuberculosis is a widespread infectious disorder affecting animals as well as humans. A major cause of this infection is a slow-growing, obligatory bacterium, which exists inside the cells, *Mycobacterium bovis*. This microbe is referred to as a well-adapted and “successful” pathogen. Its distribution is global, and several countries have been affected by its devastation in terms of economic losses and reduced herd health at livestock farms [1]. Many advanced countries have opted for the use of pasteurization in order to reduce the spread of infection, but the disease continues to cause economic/production losses when poorly controlled. The Office International des Epizooties categorized bTB as a List-B disease, a disease which has been declared as major public health concern over the last decade and affects the socioeconomic status of local farmers and animal breeders. It also bears a significant impact on the animal trading and export of animal goods [2, 3]. In underdeveloped countries like Africa, *M. bovis* infection has been reported in a wide range of animal species [4]. Bovine TB is also one of the major zoonotic diseases in Pakistan. The prevalence of bovine TB in buffaloes in the country has been reported from 0.51% to 12.72% [5]. In Pakistan and India, the incidence of bTB in cattle and buffalo was found in about 2.25% of the population in 1969 and 10% in 1975. In some countries, human disease caused by *M. bovis* is merely reported as TB to avoid inquiries from disease control departments, which might produce problems of patient privacy [6]. Transmission of *Mycobacterium bovis* in animal herds is usually via inhalation and ingestion [7]. Resistance to infection could be mediated either by the innate or adaptive immune system, and, therefore, the genomic regions related to either of these processes may be considered as candidate genes for bTB susceptibility loci [7]. IFNg is clearly an imperative cytokine in the control of the infection largely due to its potent role in macrophage activation [8–11] and is one of the major responders in *Mycobacterium* infections.

The article "Exploring the Potential of Interferon Gamma Gene as Major Immune Responder for Bovine Tuberculosis in River Buffalo" was retracted in 2024. Reasons: signs of a paper mill; suspected computer-generated content; unreliable results or conclusions; concerns about the data.

The aim of the study provides evidence in the progression of bovine tuberculosis to clinical stages is associated with reduced expression of IFNg at the site of infection. Bovine IFNg is the major gene involved in the production of IFNg, a cytokine involved in delayed type of hypersensitivity response in buffalo. In the present study, candidate polymorphisms in IFNg gene that play a part in the immunologic response were identified. Hardy Weinberg equilibrium and chi^2^ testing depicted the significance of each locus in a population. Association testing was performed to evaluate the significance of each locus with bTB susceptibility. Network and pathway analyses were also performed. Finally, protein structural configuration was studied to evaluate the genomic closeness with other bovine species. Results of this study illustrate the uniqueness of the genomic architecture of IFNg in Pakistani river buffalo, and identified polymorphisms provide a better understanding of superior animal selection that confers immunity against bTB.

## 2. Materials and Methods

This study was conducted to explore the novel SNPs in the exonic regions of IFNg, which affect the immunologic status of the buffalos that ultimately leads to the resistance or susceptibility of bovine TB in buffalo. This research work was conducted at the Postgraduate Genomics lab, Institute of Biochemistry and Biotechnology, University of Veterinary and Animal Sciences (UVAS), Lahore. This study has been approved by the University of Veterinary and Animal Sciences Research Ethics Committee and has been performed in accordance with the ethical standards.

### 2.1. Animals Selection Criteria

A clutch of 50 animals (buffalos) with specific phenotypic features for the Nili-Ravi buffalo breed were selected from different relative herds with their Bovine TB status records from UVAS Pattoki campus, Research Farm B, and Buffalo Research Institute (BRI) Pattoki. These 50 animals were bifurcated into two heads for the purpose of blood sampling, each group consisting of 25 animals. The two groups were as follows:

1. Nili Ravi buffalo showing positive skin tuberculin test and Physical features
2. Nili Ravi buffalo with negative skin tuberculin test and no previous history of lung infection

The characterization of the Positive bTB animals was done on the basis of certain phenotypic parameters as emaciation, prominent transverse process, sharped neural spines, dorsal spines individually pointed to the touch and hips, pins, tail-head, and ribs were eminent. Scoring system proposed for gross pathologic condition was used as proposed by [12]. This scoring system was based on the lesions in viscera specially lungs. Lesions were scored for caseous necrosis, mineralization, cavitation, granuloma formation, etc. In this system, varying degrees of lesions from firm or hard white, grey, or yellow nodule with a yellow, caseous, necrotic center, which was dry and solid to thin-walled suppurative abscesses were categorized as postmortem positive Elizabeth et al.1996. Detail is mentioned in Tables 1(a) and 1(b).

### 2.2. Sampling Strategy

The blood sampling of mentioned animal groups (based on the phenotypic expression of anatomical signs antemortem and postmortem scoring) was carried out. Animals group (*n* = 25) without these lesions was classified as postmortem negative.

### 2.3. Blood Sampling

Observing standard operating procedures blood samples were drawn from the jugular vein into a 50 ml falcon tube containing 200 gl of anticoagulant, i.e., EDTA (ethylene diamine tetra—acetic acid).

The article "Exploring the Potential of Interferon Gamma Gene as Major Immune Responder for Bovine Tuberculosis in River Buffalo" was retracted in 2024. Reasons: signs of a paper mill; suspected computer-generated content; unreliable results or conclusions; concerns about the data.

### 2.4. Genomic DNA Extraction/Quantification

DNA extraction was done by using standard organic method using phenol-chloroform, isoamyl alcohol (Sambrook and Russell, 2001) [13], and quantification was done by using NanoDrope Spectrophotometer and 0.8% agarose gel electrophoresis.

### 2.5. Genetic Characterization of IFNg Gene

Interferon-gamma in bovine species is located on chromosome 5. It has 4 exons with a total length of 2743 bp. Genomic characterization was done by designing specific primers to amplify the various regions of the gene by using Primer3 software (http://frodo.wi.mit.edu/) and using the sequence reported in the NCBI database (https://www.nlm.nih.gov) (Table 2).

### 2.6. Amplification and Sequencing the PCR Products

Primers were optimized and amplified on specific annealing temperature and PCR reaction mixture. PCR products were precipitated by using ethanol and sequenced using the ABI Genetic analyzer 3130 XL (Applied Biosystems, USA).

### 2.7. Bioinformatics Analysis

Sequences were aligned by using ClustalW, Multiple Alignment Tool (https://www.genome.jp/tools-bin/clustalw). Protein structural configuration of IFNg in *Bos taurus* and Nili-Ravi buffalo was created by using Phyre2 software (http://www.sbg.bio.ic.ac.uk/). Further pathway analysis was of IFNg in tuberculosis disease pathway was performed through KEGG (https://www.genome.jp/kegg/pathway.html), and network analysis of IFNg in *Bos taurus* and Nili-Ravi buffalo was carried out using STRING (ver. 11.0) knowledgebase resource (https://string-db.org/).

### 2.8. Statistical Analysis

Evaluation of the difference between allelic and genotypic frequency of the gene under study was done by using chi-square test and association analysis through calculating the odds ratio using SHEsis (http://analysis.bio-x.cn).

## 3. Results

The purpose of this study was to identify the effect of single nucleotide polymorphisms in the interferon-gamma gene in Nili Ravi buffalo. Different statistical and bioinformatics tools were used to analyze the genetic variations.

### 3.1. Statistical Significance of Data

A total of eight SNPs (single nucleotide polymorphisms) were identified in the coding region of IFNg. Among all the eight SNPs identified, four were transitions (*p*.274*G* > *A*, *p*.294 *T* > *C*, *p*.336*G* > *A*, and *p*.342 *T* > *C*) and remaining were transversions (*p*.264*G* > *C*, *p*.433 *T* > *A*, *p*.1441*A* > *C*, and *p*.1545*G* > *C*) (Table 3). *p*.294 *T* > *C* and *p*.433 *T* > *A* were nonsignificant (*P* < 0.05) and were obeying Hardy Weinberg Equilibrium (HWE). *p*.294 *T* > *C* was observed having the highest value for chi2; 0.243009 (>0.05). This variation is a potentiated marker for single locus association analysis and further selection in the breeding program. The remaining all were significantly deviating from HWE. The lowest chi^2^ score was observed for *p*.1545*G* > *C* (0.000111 < 0.05) (Table 3).

The article "Exploring the Potential of Interferon Gamma Gene as Major Immune Responder for Bovine Tuberculosis in River Buffalo" was retracted in 2024. Reasons: signs of a paper mill; suspected computer-generated content; unreliable results or conclusions; concerns about the data.

Allelic frequencies were also calculated for all loci (Table 4). The frequency range for allele-A was from 0.2097 to 0.9137, while for allele-B was from 0.0863 to 0.7903. Shannon index was also calculated for all variations depicting the gene diversity for all loci. The range of the *I*-score was 0.1937 to 0.6743, indicating the lower to medium diversity of this gene in river buffalo (Table 5).

Heterozygosity statistics were also calculated indicating the expected and observed heterozygosity of each locus. The average score of gene heterozygosity was 0.3245 with a standard deviation of 0.2093 (Table 6). Haplotypes were constructed by blocking the genomic variations. The odds ratio was calculated with a confidence interval (CI) of 95%, and maximum score observed was 2.667 with chi^2^ value 0.007 (Table 7). This indicated the significance of these variations to move together into the next generation.

### 3.2. Bioinformatics Significance of the Data

Bioinformatics analysis was done to construct a three-dimensional protein structural model and secondary structure prediction (Figure 1). It was observed that the numbers of residues were the same in Nili-Ravi buffalo and *Bos taurus* protein of IFNg. The structural model of both species did not show significant variation. Both models were carrying *α*–Helix and *β*-sheets. A significant variation in structural configuration was observed in Nili-Ravi buffalo in the form of a transmembrane helix between residues 66-81 directing from extracellular matrix to cytoplasmic medium (Figure 2). This helix could not be predicted in the 3-D structure of IFNg protein in *Bos taurus*. Pathway analysis in tuberculosis revealed that IFNg inhibits the antigen-presenting cells (APC) through JAK and STAT pathways (Figure 3). No difference in pathways of IFNg mediated inhibition of APC was found in *B. Taurus and B. Bubalis.* Network analysis of IFNg proteins in both species showed strong associations among the immunity-related proteins (interleukins, tissue necrosis factors) and receptors of interferons (Figure 4).

## 4. Discussion

The bacterium, Mycobacterium bovis, causes chronic respiratory disease and has a major impact on the cattle and buffalo industry worldwide as well as posing a risk to humans and other animal populations. In Punjab (Pakistan), the prevalence of bovine tuberculosis varies in buffaloes from 12.48% to 33.72% [14]. Despite over sixty years of costly eradication programs, including the vaccination, regular monitoring at farms, and periodic slaughter of infected animals, the number of cases continues to rise. According to Health Department, Government of Punjab, Pakistan is ranked 8th among the 22 high tuberculosis burdened countries in the world and about 300,000 new cases are added each year. There are also issues like drug residues in animal products and drug resistance by the pathogens that demand new control strategies for this infection. Previous studies have suggested that animals differ genetically in their risk of bovine tuberculosis. This has opened up the possibility of breeding animals that have a lower risk of becoming infected with bovine tuberculosis. Colin [15] and his team provided the first hand report about the genetic basis to natural resistance to infections such as bovine tuberculosis, with an estimated heritability of 0.48 (standard error, 0.096; *P* < 0.01). The breeding of selection lines of resistant and susceptible animals provided an ideal strategy for reducing the number and severity of outbreaks of Tb in farmed animals. Identifying candidate genes and novel polymorphisms are crucial to economically important infectious diseases, which ultimately can provide a method for the selection of resistant animals in a more targeted and efficient way. But this solution is a long-term one and needs extensive research. Previous studies have suggested that animals differ genetically in their risk of bovine tuberculosis [16–18]. This has opened up the possibility of breeding animals, which have a lower risk of becoming infected with bovine tuberculosis.

The article "Exploring the Potential of Interferon Gamma Gene as Major Immune Responder for Bovine Tuberculosis in River Buffalo" was retracted in 2024. Reasons: signs of a paper mill; suspected computer-generated content; unreliable results or conclusions; concerns about the data.

In this context, this study was planned for genetic screening of the Interferon-gamma gene in the Nili Ravi buffalo of Pakistan. A total of eight SNPs were identified in the coding region of the IFNg gene. The one SNP found in the current research is in compliance with the research on IFNg, hence, seven SNPs found in the current research are novel in Nili Ravi buffalo. SNPs in the IFNg gene have also been reported by [19] and considered as candidate markers for controlling the Bovine Tuberculosis in Chinese Holstein cattle.

For the analysis of population, genetics at all the loci POPGENE 32 software was used. By using this software, overall allele frequency, heterozygosity, probability using Chi-square test, and Likelihood ratio test Hardy-Weinberg equilibrium, gene diversity of all SNP position was calculated.

The results of the study follow the postulates of the Hardy-Weinberg equilibrium demonstrating that the two of the identified alleles were randomly distributed throughout the population, no migration had occurred, no bottlenecks happened, and the population remained large in numbers. These nonsignificant variations were obeying HWE and can be potential markers for genetic selection. Polymorphisms with a probability value below 0.05 indicated that the population at these polymorphic sites was not obeying Hardy-Weinberg equilibrium. This indicated that at these positions, alleles were not equally distributed in population.

The article "Exploring the Potential of Interferon Gamma Gene as Major Immune Responder for Bovine Tuberculosis in River Buffalo" was retracted in 2024. Reasons: signs of a paper mill; suspected computer-generated content; unreliable results or conclusions; concerns about the data.

The mean value of effective number of alleles (ne) was 1.59522, and the mean value score for the observed number of alleles (na) was 2.0000, which is higher than (ne) demonstrating that Mutant alleles are more in the animal population, which could not pass on to the next generation as a whole. The mean value of observed homozygosity and observed heterozygosity was 0.8900 and 0.1100. Similarly, expected homozygosity and heterozygosity mean were 0.6584 and 0.3416, respectively. The average heterozygosity mean value was 0.3245 ± 0.2093 (SD).

3-D protein structure of IFNg protein in buffalo and cattle was compared, and unique secondary structures were observed. A transmembrane helix was predicted in buffalo, which was missing in the cattle IFNg protein of cattle. Moreover, it is also revealed that IFNg inhibits the antigen-presenting cells (APC) through JAK and STAT pathways in tuberculosis disease [9, 11].

## 5. Conclusion

It can be concluded from the above discussion that the polymorphisms in the IFNg gene are likely to be involved in susceptibility to bovine tuberculosis. The IFNg gene may also carry the potential for Marker-assisted breeding uses DNA markers associated with desirable traits to select an animal for inclusion in a breeding program early in its development and eyeing for BTB-resistant animals within both the national farms and the private sector. The outcomes of this study are aimed at generating baseline information about the genomic markers for our indigenous river buffalo for improvement of its genetic potential against bovine tuberculosis.

## Figures and Tables

**Figure 1:** 3-D protein structural configuration of IFNg protein in Nili Ravi Buffalo and *Bos taurus.*

**Figure 2:** Transmembrane loop identified in IFNg protein of Nili Ravi buffalo.

**Figure 3:** KEGG Pathway analysis of IFNg protein in tuberculosis disease. The role of IFNg is represented in the inhibition of antigen-presenting cells through the JAK and STAT pathways.

**Figure 4:** Network analysis of IFNg protein of (a) *B. Taurus* and (b) *Nili Ravi buffalo* using STRING knowledgebase (11.0 Ver.).

**Table:** (a) Description of condition scores for Positive samples

Score	Condition	Features (antemortem)	(Postmortem)	PPD^∗^
1	L-	Marked emaciation	Caseous necrosis	+ve
2	L	Transverse processes project prominently, neural spines appear sharply.	Mineralization	+ve
3	L+	Individual dorsal spines are pointed to the touch; hips, pins, tail-head, and ribs are prominent. Transverse processes visible, usually individually	Cavitation	+ve

^∗^Purified protein derivative.

The article "Exploring the Potential of Interferon Gamma Gene as Major Immune Responder for Bovine Tuberculosis in River Buffalo" was retracted in 2024. Reasons: signs of a paper mill; suspected computer-generated content; unreliable results or conclusions; concerns about the data.

**Table:** (b) Description of condition scores for negative samples

Score	Condition	Features (antemortem)	(Postmortem)	PPD
1	F-	Animal smooth and well covered, but fat deposits are not marked. Dorsal spines can be felt with firm pressure, but feel rounded rather than sharp.	No lesion	-ve
2	F	Fat cover in critical areas can be easily seen and felt; transverse processes cannot be seen or felt.		-ve
3	F+	Heavy deposits of fat clearly visible on tail-head, brisket, and cod; dorsal spines, ribs, hooks, and pins fully covered and cannot be felt even with firm pressure.		-ve

**Table 2:** IFNg gene primers.

Sr. no.	Primer names	5′-3′ sequences
1	IFNG1 (F)	5–ccagcaccaaaaggagacac-3
	IFNG1 (R)	5-gaagactagagatgagagccca-3
2	IFNG2 (F)	5-gtgccagcatccaagttcaa-3
	IFNG2 (R)	5-agcaacaggaaaatcagccaa-3
3	IFNG3 (F)	5-tcctaatgactcataggcctga-3
	IFNG3 (R)	5-tgtttcatttaacccagcccc-3

**Table 3:** SNPs identified in IFNg in Nili Ravi buffalo.

SNP	Location	Wild	Mutant	Transition/ transversion	Chi^2^ (<0.05)	HWE
*p*.264*G* > *C*	45830264	G	C	Transversion	0.040418	S^∗^
*p*.274*G* > *A*	45830274	G	A	Transition	0.033603	S
*p*.294 *T* > *C*	45830294	T	C	Transition	0.243009	NS^∗^
*p*.336*G* > *A*	45830336	G	A	Transition	0.000649	S
*p*.342 *T* > *C*	45830342	T	C	Transition	0.000262	S
*p*.433 *T* > *A*	45830433	T	A	Transversion	1.000000	NS
*p*.1441*A* > *C*	45831441	A	C	Transversion	0.015112	S
*p*.1545*G* > *C*	45831545	G	C	Transversion	0.000111	S

^∗^S: significant. ^∗^NS: nonsignificant.

**Table 4:** Allele frequency of multiple loci identified in IFNg in Nili Ravi buffalo.

Allele/locus	Allele A	Allele B
*p*.264*G* > *C*	0.3030	0.6970
*p*.274*G* > *A*	0.7523	0.2477
*p*.294 *T* > *C*	0.3733	0.6267
*p*.336*G* > *A*	0.3939	0.6061
*p*.342 *T* > *C*	0.6371	0.3629
*p*.433 *T* > *A*	0.2097	0.7903
*p*.1441*A* > *C*	0.5432	0.4568
*p*.1545*G* > *C*	0.9137	0.0863

**Table 5:** Shannon index of genomic variations in IFNg gene depicting diversity.

Locus	Sample size	na^∗^	ne^∗^	I
*p*.264*G* > *C*	50	2.0000	1.9231	0.6595
*p*.274*G* > *A*	50	2.0000	2.0000	0.6743
*p*.294 *T* > *C*	50	2.0000	1.6000	0.6288
*p*.336*G* > *A*	50	2.0000	2.0000	0.5710
*p*.342 *T* > *C*	50	2.0000	1.7241	0.1937
*p*.433 *T* > *A*	50	2.0000	1.1050	0.6402
*p*.1441*A* > *C*	50	2.0000	1.6000	0.6743
*p*.1545*G* > *C*	50	2.0000	1.0000	0.5823

The article "Exploring the Potential of Interferon Gamma Gene as Major Immune Responder for Bovine Tuberculosis in River Buffalo" was retracted in 2024. Reasons: signs of a paper mill; suspected computer-generated content; unreliable results or conclusions; concerns about the data.

**Table 6:** Summary of heterozygosity statistics of IFNg in Nili Ravi Buffalo.

Locus	Obs_Hom	Obs_Het	Exp_Hom^∗^	Exp_Het^∗^	Nei^∗∗^	Ave_Het
*p*.264*G* > *C*	0.8000	0.2000	0.4947	0.5053	0.4800	0.4800
*p*.274*G* > *A*	0.8000	0.2000	0.4737	0.5263	0.5000	0.5000
*p*.294 *T* > *C*	0.5000	0.5000	0.6053	0.3947	0.3750	0.3750
*p*.336*G* > *A*	1.0000	0.0000	0.4737	0.5263	0.5000	0.5000
*p*.342 *T* > *C*	1.0000	0.0000	0.5579	0.4421	0.4200	0.4200
*p*.433 *T* > *A*	0.9000	0.1000	0.9000	0.1000	0.0950	0.0950
*p*.1441*A* > *C*	0.9000	0.1000	0.6053	0.3947	0.3750	0.3750
*p*.1545*G* > *C*	1.0000	0.0000	1.0000	0.0000	0.0000	0.0000
Mean	0.8900	0.1100	0.6584	0.3416	0.3245	0.3245
St. dev	0.1595	0.1595	0.2203	0.2203	0.2093	0.2093

**Table 7:** Association analysis of haplotypes by calculating odds ratio in IFNg gene.

Haplotype	Chi^2^	Pearson's *P*	Odds ratio (95% CI)
A B A A B B B A	0.916	0.338615	—
A B B A B B B A	0.007	0.931562	1.133
A B B B B B B A	0.036	0.931562	1.133
B B A A B B B B	0.094	0.848878	1.167
B B B A B B B A	0.007	0.289049	2.667
B B B B A B B A	0.916	0.122060	—

## Data Availability

This study's data will be available openly to readers and can access the data supporting the conclusions of the study.
